# Day-ahead electricity price forecasting using WPT, VMI, LSSVM-based self adaptive fuzzy kernel and modified HBMO algorithm

This article has been retracted.

**DOI:** 10.1038/s41598-021-96501-6

**Published:** 2021-08-30

**Authors:** Rahmad Syah, Mohammad Rezaei, Marischa Elveny, Meysam Majidi Nezhad, Dadan Ramdan, Mehdi Nesaht, Afshin Davarpanah

**Affiliations:** 1 Data Science & Computational Intelligence Research Group, Universitas Medan Area, Medan, Indonesia; 2 Computer Science and Engineering Department, University of Texas at Arlington, Arlington, USA; 3 Data Science & Computational Intelligence Research Group, Universitas Sumatera Utara, Medan, Indonesia; 4 Department of Astronautics, Electrical and Energy Engineering (DIAEE), Sapienza University of Rome, 00184 Rome, Italy; 5 DS & CI Research Group, Universitas Medan Area, Medan, Indonesia; 6 Optimisation and Logistics Group, School of Computer Science, University of Adelaide, Adelaide, Australia; 7 Department of Mathematics, Aberystwyth University, Aberystwyth, SY23 3FL UK

**Keywords:** Energy grids and networks, Electrical and electronic engineering

## Abstract

Due to focal liberality in electricity market projection, researchers try to suggest powerful and successful price forecasting algorithms. Since, the accurate information of future makes best way for market participants so as to increases their profit using bidding strategies, here suggests an algorithm for electricity price anticipation. To cover this goal, separate an algorithm into three steps, namely; pre-processing, learning and tuning. The pre-processing part consists of Wavelet Packet Transform (WPT) to analyze price signal to high and low frequency subseries and Variational Mutual Information (VMI) to select valuable input data in order to helps the learning part and decreases the computation burden. Owing to the learning part, a new Least squares support vector machine based self-adaptive fuzzy kernel (LSSVM-SFK) is proposed to extract best map pattern from input data. A new modified HBMO is introduced to optimally set LSSVM-SFK variables such as bias, weight, etc. To improve the performances of HBMO, two modifications are proposed that has high stability in HBMO. Suggested forecasting algorithm is examined on electricity markets that has acceptable efficiency than other models.

## Introduction

In this section, we state the issue and goals in this article. To create a more orderly structure, the introduction is divided into the following sections.

### Important of price forecasting

Over the recent years, modern technologies^1–5^ shows more potential as view of electricity industry relaxation^6–10^ which leads to clear market without an extra force^11–26^, therefore, the number of market participants is increased since they freely accessed to market information^1–9^. Owing to the participants growing and the intense competition forces, the first, fast and correct decisions will be necessary for both enterprises and academia to maximize profit which itself needed to more accurate information of electricity price^27–41^. Owing to the uneconomical way for energy storage^42–47^ in large-scale and its decency to different factors such as holidays^48–52^, sudden disturbance in transmission and generation power systems, celebrations, season, etc.^53–55^. the electricity price forecasting will be more difficult than any other financial markets^56–63^. In other words, electricity markets price are the result of the intersection of supply and demand curves^64–70^. The supply demand directly affects by weather conditions and general economy behaviors. In supply side, prices of fuel i.e. gas, coal, oil, etc. and unexpected fails also plays an important role^71–76^. As result, Fig. 1 shows a graphical view of important factors which directly affects on power prices. It is clear that these factors make fluctuations in electricity price signals.

**Figure 1:** Graphical view of electricity price which directly reflects important and effective factors in price fluctuations.

### Literature review

Recently, researchers have high difficulty for modulation of electricity prices. In according to literature, the modeling of forecasting of electricity price is arranged via 3 groups: the first group is short-term, the second group is mid-term and the third group is long-term. The mentioned 3 groups of modeling of forecasting of electricity price are presented in Fig. 2. The mid- and long-terms are beneficial to reciprocal conventions and to generate the planning. However, forecasting via short-term has high important for derivative conventions. Particularly, the forecasting of electricity price has main interest in all actions of market, daily. Due to variations of electricity price, the short-term is requested the high precision to provide the trusty intention for participants. In literature the modeling of forecasting of electricity price is arranged to classical model and intelligent model.

**Figure 2:** Three main classes of forecasting based on time horizons.

The classical group consists of ARIMA^76^, DR^77^, GARCH^78^, mixed-model^79^, transfer function model^80^ and etc. However, these methods have been popular but in modern electricity market, they need a lot of information to be accurate and usually have high computational times. Moreover, their liner structure usually raises forecast error because they can’t capture the non-liner pattern of input data. The forecasted load and day ahead weather are implemented in security-constrained unit commitment to schedule the preventive power flow^81^.

In spite of aforementioned methods, the intelligent group covers different methods based on machine learning, decomposition technique and feature selection that have been effectively employed to forecast the electricity price^82^. This group tries to combine different methods to use all potential in forecasting, therefore, hybrid methods have been generally employed in price forecasting. In Ref.^83^ proposed hybrid algorithm based on MI, WT, LSSVM and Chaotic Gravitational Search Algorithm (CGSA) for price forecasting.

Maciejowska et al.^84^ indicated that anticipation of mentioned main variables that were presented via Transmission System Operators are biased and these anticipation can be improved via ordinary regression methods. The improved predictions can use to forecast the prices of dot and within the day in Germany. Muniain et al.^85^ investigated the dependency of forecasting of electricity price and measurement. Here, we examined the series of off-peak and peak time of German-Austrian of price day. Therefore, we investigated the bi-variate information and data. We evaluated the average of time series, firstly and then we examined the residuals, secondly. The average equation is calculated via normal least squares and elastic pure and the residuals are calculated via maximum likelihood. Brusaferri et al.^86^ suggested the new model to forecast the price of energy by using of the Bayesian methods. The specific model has been extend to warranty of various network architectures. Furthermore in this study we extend a method that enduring the hetero-scedasticity. Therefore eluding the usual homo–scedastic presumption via their pre-processing attempt.

In Ref.^87^ introduced an algorithm for price forecasting by take into account a perspective on the data i.e. seasonal behavior, renewable energy. In this mythology try to use true information between the sale and purchase curves based on X-model which able to capture the nonlinear model of price spikes.

The abrupt event of some spike prices in electricity dot market is affected on accuracy of forecast of electricity price, importantly. Shi et al.^88^ suggested new 2-step scheme to forecast of electricity price (TSEP). In step one the scheme to predicate the multi-source data-based spike is proposed, that it accepted network of deep neural (DNN) for prediction whether increasing price is spike or not. Averaging of Quantile Regression (QRA) is made the high interest for forecasting of electricity price when it unique vicrory in contest 2014 for forecasting of energy, that 2 incisive teams are used the QRA variants. Even so, the recent works have presented model’s vulnerability for down quality to predict that regressor sets are greater than any. To investigate of mentioned problem, Uniejewskiet al.^89^ are chosen the normal variant of QRA, that is used Least Absolute Shrinkage and Selection Operator (LASSO) for choosing relevant regressor, automatically. In this study, mentioned techniques are examined by using of the datasets of Polish and Nordic markets of power. In this study, we prepared the document for better predictive efficiency in Kupiec, pinball mark and test for eventual accuracy by comparsion to various of benchmarks. Mainly, when ordered parameter is chosen ex-ante by using of Bayesian Information Criterion (BIC).

In Ref.^90^ proposed a generalized neuron method for electricity price forecasting of Australian electricity market. Moreover, used WT to remove noise term of electricity price and get better pattern for learning. In Ref.^91^ proposed a new hybrid algorithm based on WPT, LSSVM based Bayesian theory for day-ahead electricity price forecasting. Shorting speaking, a simple classification with general view of various forecasting methods is shown in Fig. 3. Note that this rough tree can be developed in more details and other methods may be considered as a new branch. Form on prediction factors such as: type of model, input/output variables, time horizon, pre-processing part, learning part and etc., there is problem in prediction. Goals of here is to offer an effective and prediction framework for forecasting from perspective.

**Figure 3:** A simple classification of price-forecasting methods as well as load forecasting.

### Motivation and contribution

The series of electricity price are combined from non-linear component and linear correlation construction. So, the hybrid model with abilities of linear and nonlinear modeling, it is useful strategy to forecast of price. The forecasting of price of electricity is hard due to unlike load, the series of electricity price are presented some properties such as non-constant variance, great frequency. Therefore, transferring the wavelet is utilized for convention the series of price to series constitutive, that it presented the better behavior than series of original price. So, their results are predicted with high efficiency. Consequently, the hybrid model via WT, feature election and LSSVM are suggested. The stimulation to accept the hybrid model is to usage another models’s feature to receive several patterns in series of electricity price. The theoretical and empirical results and data are proposed that combination of several models is effective and that is usual strategy to increase the accuracy of forecasts. As aforementioned illustrations, contribution of this study can be stated as follows:

- Owing to the fast growing of input data with their inherent noisy term, each learning method needs a powerful feature selection to chose best of them with least redundancy^92^. Therefore, as a contribution of this paper, proposes a Variational Mutual Information (VMI) which employed the beneficial theory of wrapping and filter models^93^. Since the electricity price has an inherent uncertainties, VMI use a new probably function with three-way feature selection based on variational distribution function and lower bound to estimate their relevancy and redundancy in more details without its dependency to MI estimating.
- Specially, the WPT is employed to decompose electricity price signal into high and low frequency terms to make better pattern for learning part. Since the created tree of WPT has high computational time, a Shannon–Renyi entropy criterion based on the probability distribution is employed to select best branches.
- As shown in next section, the kernel function plays important role to make best pattern among of input data, therefore, LSSVM-SFK is proposed. Self-adaptive fuzzy combination to LSSVM is increased day-ahead electricity price forecasting accurate.
- Albeit the HBMO has been shown an effective performance in different engineering problems^94–96^. To obtain the LSSVM-SFK potential, its variables such as penalty factor, bias and weights must be set by a powerful algorithm. Since the standard HBMO often trapped in local solutions, some modifications were suggested in HBMO and global updating.

To the reader convenience, the contribution of this paper is shown in Fig. 4.

**Figure 4:** Outline of the main contributions for this paper in day-ahead electricity price forecasting.

## Proposed price-forecasting tools

In this section, we have tried to express the tools used in the forecasting model. To create more order, each tool is described in detail in its respective subsection.

### WPT

WPT is a powerful tool to present a signal in time and frequency domain without lost any information. WPT is similar to Discrete WT (DWT) except it uses all subseries in high and low filters. In more details about DWT refer to^97^. Shorting speaking without losing the general illustrations, an estimated price signal at resolution 2-j can be defined on Vj ⊂ L2(R) which Vj consists of previous spaces to resolution 2-j. Let xj be projection of x on Vj so distance kx–xjk will be minimized. The details term coming to resolutions 2 − j + 1 and 2 − j. The approximation and details terms are shown in Fig. 5.

**Figure 5:** Presentation of approximation (*V*_*j*_) and detail spaces (*W*_*j*_) in WPT decomposing.

It is clear that the details term at resolution 2^*j*^ can be calculated by orthogonal projection in spaces *V*_*j*_ and *V*_*j−1*_, $W_{j} \oplus V_{j} = V_{j - 1}$, and orthogonal function is $\phi_{j,n} = \frac{1}{{\sqrt {2^{j} } }}\phi \left( {\frac{{t - 2^{j} n}}{{2^{j} }}} \right)$.

All $\{ \phi_{j} (t - 2^{j} n)\}_{n \in Z}$ is obtained via $V_{j + 1} = \{ \phi_{j + 1} (t - 2^{j + 1} n)\}_{n \in Z}$ and $W_{j + 1} = \{ \varphi_{j + 1} (t - 2^{j + 1} n)\}_{n \in Z}$ which can be defined by two high (H) low (L) pass filters, one gets:

1 $$H(n) = \left\langle {\frac{\phi (0.5t)}{{\sqrt 2 }},\phi (t - n)} \right\rangle ,$$

2 $$\left\langle {\phi_{j + 1,p} ,\phi_{j,n} } \right\rangle = \left\langle {\frac{\phi (0.5t)}{{\sqrt 2 }},\phi (t - n + 2p)} \right\rangle = H(n - 2p),$$

3 $$\phi_{j + 1,p} = \sum\limits_{n \in ( - \infty , + \infty )} {H(n - 2p)\phi_{j,n} } ,$$

4 $$G(n) = \left\langle {\frac{\varphi (0.5t)}{{\sqrt 2 }},\phi (t - n)} \right\rangle ,$$

5 $$\left\langle {\varphi_{j + 1,p} ,\phi_{j,n} } \right\rangle = \left\langle {\frac{\varphi (0.5t)}{{\sqrt 2 }},\phi (t - n + 2p)} \right\rangle = G(n - 2p),$$

6 $$\varphi_{j + 1,p} = \sum\limits_{n \in ( - \infty , + \infty )} {G(n - 2p)\phi_{j,n} } ,$$

7 $$G(n) = ( - 1)^{ - n + 1} H( - n + 1).$$

As a result, the decomposition and reconstruction terms and the frequency bound are shown in Fig. 6. The main advantages responded to WPT are; (i) provides more flexible tool in high and low pass filters, (ii) use all information in details, (iii) WPT integrated feature selection makes powerful preprocessing approach.

**Figure 6:** (**a**) WPT decomposition and reconstruction tree at 3 levels, (**b**) frequency bands covered by the scaling ($\varphi$) and wavelet ($\phi$) functions.

### Shannon–Renyi entropy

One of the ultimate purposes in WPT is to avoid high computational cost time caused by WPT tree. There are several entropy approaches, among them, Shannon–Renyi entropy outcomes from the selection of the logarithmic loss distribution function and shows powerful performance based on entropy to investigation branches contributions in WPT tree. For discrete variable $\mathop Y\limits^{ \to } = y_{1} ,...,y_{N}$ with probability *p*, Shannon entropy can be defined by:

8 $$H(\vec{Y}) = - E_{y} [\log (p(\vec{Y}))] = - \sum\nolimits_{i = 1}^{N} {p(\vec{Y} = y_{i} )} \log p(\vec{Y} = y_{i} ).$$

As a generalized model of Shannon entropy with Renyi *α*-entropy, one gets:

9 $$H_{\alpha } (\vec{Y}) = \frac{1}{1 - \alpha }\log \sum\nolimits_{i = 1}^{n} {y_{i}^{\alpha } } .$$

This entropy can be cover Shannon entropy models when its order *α* tends to 1.

The SVM as a learning machine is investigated by Vapnik in 1995 and shows effective performance in different researches^98^. However, the standard SVM has a difficulty in nonlinear term. In other words, in noisy signals such as electricity price, the nonlinear term has main role for learning. To cope with this aim, this paper employed LSSVM to develop nonlinear term based on least square formulation ($\sum\nolimits_{i = 1}^{l} {e_{i}^{2} }$). Shorting speaking; let $D = \left\{ {\left( {{\mathbf{x}}_{i} ,y_{i} } \right)} \right\}_{i = 1}^{l}$ is data that ${\mathbf{x}}_{i} \in R^{n}$ and $y_{i} \in \left\{ { \pm 1} \right\}$ are feature vector and the regression accuracy, respectively. The training process can be defined by:

10 $$\min J\left( {w,e} \right) = \frac{1}{2}{\mathbf{w}}^{T} {\mathbf{w}} + \gamma \frac{1}{2}\sum\nolimits_{i = 1}^{l} {e_{i}^{2} } \,{\text{s}}.{\text{t}}.\,y_{i} \left( {{\mathbf{w}}^{T} \phi \left( {{\mathbf{x}}_{i} } \right) + b} \right) = 1 - e_{i} , \, i = 1, \ldots ,l,$$

$\left( {{\mathbf{w}}^{T} \phi \left( {{\mathbf{x}}_{i} } \right) + b} \right) = y_{i} - e_{i}$ is limited algorithm form on regression error. The Lagrangian of LSSVM is obtained via:

11 $$L\left( {{\mathbf{w}},{\mathbf{e}},b;{{\varvec{\upalpha}}}} \right) = \frac{1}{2}{\mathbf{w}}^{T} {\mathbf{w}} + \gamma \frac{1}{2}\sum\nolimits_{i = 1}^{l} {e_{i}^{2} } - \sum\nolimits_{i = 1}^{l} {\alpha_{i} \left[ {\left( {{\mathbf{w}}^{T} \phi \left( {{\mathbf{x}}_{i} } \right) + b} \right) - y_{i} + e_{i} } \right]} .$$

According to KKT conditions, Eq. (11) is solved via:

12 $$\left\{ {\begin{array}{*{20}l} {\frac{{\partial L\left( {{\mathbf{w}},{\mathbf{e}},b;{{\varvec{\upalpha}}}} \right)}}{{\partial {\mathbf{w}}}} = 0 \Rightarrow {\mathbf{w}} = \sum\limits_{i = 1}^{l} {\alpha_{i} \varphi \left( {{\mathbf{x}}_{i} } \right)} } \hfill \\ {\frac{{\partial L\left( {{\mathbf{w}},{\mathbf{e}},b;{{\varvec{\upalpha}}}} \right)}}{\partial b} = 0 \Rightarrow \sum\limits_{i = 1}^{l} {\alpha_{i} } = 0} \hfill \\ {\frac{{\partial L\left( {{\mathbf{w}},{\mathbf{e}},b;{{\varvec{\upalpha}}}} \right)}}{{\partial {\mathbf{e}}}} = 0 \Rightarrow \alpha_{i} = \gamma e_{i} } \hfill \\ {\frac{{\partial L\left( {{\mathbf{w}},{\mathbf{e}},b;{{\varvec{\upalpha}}}} \right)}}{{\partial {{\varvec{\upalpha}}}}} = 0 \Rightarrow {\mathbf{w}}^{T} \varphi \left( {{\mathbf{x}}_{i} } \right) + b - y_{i} + e_{i} = 0} \hfill \\ \end{array} } \right..$$

This optimization problem is corresponding to solve the following matrix:

13 $$\left[ {\begin{array}{*{20}c} {{\mathbf{K}}_{l} + \gamma^{ - 1} {\mathbf{I}}} & {\mathbf{1}} \\ {{\mathbf{1}}^{T} } & 0 \\ \end{array} } \right]\left[ {\begin{array}{*{20}c} {{\varvec{\upalpha}}} \\ b \\ \end{array} } \right] = \left[ \begin{gathered} {\mathbf{y}} \hfill \\ 0 \hfill \\ \end{gathered} \right],$$

where $$K_{l} = \left[ {k_{ij} } \right]_{i,j = 1}^{l}$$ and $$k_{ij} = k\left( {{\mathbf{x}}_{i} ,{\mathbf{x}}_{j} } \right) = \left\langle {\varphi \left( {{\mathbf{x}}_{i} } \right),\varphi \left( {{\mathbf{x}}_{j} } \right)} \right\rangle$$ are kernel. The kernel function $$k\left( {{\mathbf{x}}_{i} ,{\mathbf{x}}_{j} } \right) = \left\langle {\varphi \left( {{\mathbf{x}}_{i} } \right),\varphi \left( {{\mathbf{x}}_{j} } \right)} \right\rangle$$ is used to make better learning pattern between inputs and training vector without clearly knowing the function $$\varphi \left( {\mathbf{x}} \right)$$. There are some well-known kernel functions $$k\left( {{\mathbf{x}}_{i} ,{\mathbf{x}}_{j} } \right) = \exp \left( {{{\left\| {{\mathbf{x}}_{i} - {\mathbf{x}}_{j} } \right\|_{2}^{2} } \mathord{\left/ {\vphantom {{\left\| {{\mathbf{x}}_{i} - {\mathbf{x}}_{j} } \right\|_{2}^{2} } {2\sigma^{2} }}} \right. \kern-\nulldelimiterspace} {2\sigma^{2} }}} \right)$$ with variance $$\sigma$$, linear kernel $$k\left( {{\mathbf{x}}_{i} ,{\mathbf{x}}_{j} } \right) = {\mathbf{x}}_{j}^{T} {\mathbf{x}}_{i}$$, polynomial kernel of degree *d* and etc. Based on aforementioned kernel functions, it can be result that there is a gap to optimally choice best one. It is worth pointing out that how select the best kernel function needs many aspects such as input data and its nonlinearity. Since the fuzzy theory shows good performance without knowing previous-knowledge of system, it motivates to adopt LSSVM with fuzzy kernel to process non-linear separable data and enhance prediction ability. Let $$\rho_{ik,t} = (\mu_{ik,t} )^{{g_{t} }} ,g_{t} = (g_{0} t_{\max } - (g_{0} - 1)t)t_{\max }^{ - 1}$$ and $$\mu_{ik,t} = (||x_{k} - w_{i,t - 1} ||^{2} )^{{\frac{1}{1 - g}}} \times \sum\nolimits_{j} {(||x_{k} - w_{j,t - 1} ||^{2} )^{{\frac{1}{g - 1}}} }$$ be the learning rate and membership functions which $$g_{0} \ge 1$$, *t* and *t*_*max*_ denotes current and maximum iteration, *x*_*k*_ is *k*^*it*^ sample in class *c* which will be limited by $$\mu_{ik,t} \in [0,1]$$$$|\sum\nolimits_{i = 1}^{c} {\mu_{ik,t} = 1}$$ and $$0 < \sum\nolimits_{k = 1}^{n} {\mu_{ik,t} } < n$$. As aforementioned note, the kernel function resulting of inner product of mapping function $$\left\langle {\varphi \left( {{\mathbf{x}}_{i} } \right),\varphi \left( {{\mathbf{x}}_{j} } \right)} \right\rangle$$, hereby, the final goal is making the updating formulation for this function, one gets^99^:

14 $$J(w;x) = \arg \min ||\phi (x_{k} ) - \phi (w_{i} )||^{2} , \, w_{i,t} = w_{i,t - 1} + \frac{{\sum\nolimits_{k} {\rho_{ik,t} (x_{k} - w_{i,t - 1} )} }}{{\sum\nolimits_{j} {\rho_{ij,t} } }}.$$

According to Euclidean distance, this function can be rewrite by:

15 $$\begin{aligned} ||\phi (x_{k} ) - \phi (w_{i} )||^{2} = & (\phi (x_{k} ) - \phi (w_{i} ))^{T} \cdot (\phi (x_{k} ) - \phi (w_{i} )) = \phi (x_{k} )^{T} .\phi (x_{k} ) - \phi (x_{k} )^{T} \phi (w_{i} ) \\ & - \phi (w_{i} )^{T} .\phi (x_{k} ) = \left\langle {\phi (x_{k} ),\phi (x_{k} )} \right\rangle + \left\langle {\phi (w_{i} ),\phi (w_{i} )} \right\rangle - 2\left\langle {\phi (x_{k} ),\phi (w_{i} )} \right\rangle . \\ \end{aligned}$$

Then, the membership functions can be updated by:

16 $$\mu_{ik,t} = \frac{{[K(x_{k} ,x_{k} ) + K(w_{i} ,w_{i} ) - 2K(x_{k} ,w_{i} )]^{{\frac{1}{1 - m}}} }}{{\sum\nolimits_{p = 1}^{c} {[K(x_{k} ,x_{k} ) + K(w_{p} ,w_{p} ) - 2K(x_{k} ,w_{p} )]^{{\frac{1}{1 - m}}} } }}.$$

Substituting Eq. (16) in $\rho_{ik,t} = (\mu_{ik,t} )^{{g_{t} }}$, then learning rate will be updated.

### Variational mutual information (VMI)

Feature selection was utilized approach to choose relevant feature subset for successful classification or regression of data. Especially, in high-dimensional input data, the performance of a classifier or predictor directly depends on the feature subset^100^. This section focused on proposed VMI, interested reader can refer to^100^ for basic formulation of mutual information which is main background of VMI. Usually, high-dimensional data has an inherent difficulty to estimate their relevancy. Therefore, mutual information has been developed in low-order approximation;

$\mathop {\arg \max }\limits_{{i \notin C^{t - 1} }} I(x_{i} ,y) + H(x_{{C^{t - 1} }} |x_{i} ) - H(x_{{C^{t - 1} }} |x_{i} ,y)$ which *X* = *{x*_1_, *x*_2_,…, *x*_*n*_*}* is input data, ***y*** is training vector and *C* is best class with most relevancy. In order to have an exact estimate of $H(x_{{C^{t - 1} }} |x_{i} ) \approx \sum\nolimits_{k = 1}^{t - 1} {H(x_{{f_{k} }} |x_{i} )}$ and $H(x_{{C^{t - 1} }} |x_{i} ,y) \approx \sum\nolimits_{k = 1}^{t - 1} {H(x_{{f_{k} }} |x_{i} ,y)}$^93^, there have two assumptions; (i) Independence features $p(x_{{C^{t - 1} }} |x_{i} ) = \mathop \prod \limits_{k = 1}^{t - 1} p(x_{{f_{k} }} |x_{i} )$ and (ii) Class-conditioned independence $p(x_{{C^{t - 1} }} |x_{i} ,y) = \mathop \prod \limits_{k = 1}^{t - 1} p(x_{{f_{k} }} |x_{i} ,y)$. These assumptions show that *x*_*i*_ is independent or class-conditionally independent, respectively. If variable ***x***_*i*_ with training variable ***y*** have joint distribution function *p*(***x***_*i*_*; ****y***) and arbitrary variational distribution *q*(***x***_*i*_*|****y***), the lower-bound of MI can be defined by^101^:

17 $$I(x_{i} ,y) \ge H(x_{i} ) + mean(\ln q(x_{i} |y))_{{p(x_{i} ,y)}} ,\sum\nolimits_{x} {p(x_{i} |y)\log \frac{{p(x_{i} |y)}}{{q(x_{i} |y)}} \ge 0} .$$

Note that this bound will be exact if $p(x_{i} |y) \equiv q(x_{i} |y)$. Main goal of VMI is optimize the lower bound in optimal class C^*^ by:

18 $$C^{*} = \mathop {\arg \max }\limits_{C} \{ H(x_{C} ) + mean(\ln q(x_{C} |y))_{{p(x_{C} ,y)}} \} .$$

According to aforementioned illustrations, the lower bound can be rewrite by:

19 $$I(x_{C} :y) \ge H(y) + mean(\ln q(x_{C} |y))_{{p(x_{C} ,y)}} = mean(\ln (\frac{{q(y|x_{C} )}}{p(y)}))_{{p(x_{C} ,y)}} ,if \, H(y) = mean( - \ln p(y))_{p(y)} .$$

Therefore, the final lower bound can be calculated by:

20 $$C^{*} = \mathop {\arg \max }\limits_{C} \left\{ {mean(\ln (\frac{{q(y|x_{C} )}}{p(y)}))_{{p(x_{C} ,y)}} } \right\}.$$

where $q(y|x_{C} )$ is a normalized distribution function, one gets:

21 $$q(y|x_{C} ) = \frac{{q(x_{C} ,y)}}{{q(x_{C} )}} = \frac{{q(x_{C} |y)p(y)}}{{\sum\nolimits_{{y^{\prime}}} {q(x_{C} |y^{\prime})p(y^{\prime})} }}.$$

Resulting, the lower bound is $I(x_{C} :y) \ge mean(\ln (\frac{{q(x_{C} |y)}}{{q(x_{C} )}})) \equiv I_{LB} (x_{C} :y)$. Generally speaking, the final feature selection in three ways can be expressed as follows:

22 $$VMI = \arg \max \left( {I(x_{i} ;C^{*} ) + \mathop {\min }\limits_{{X_{s} \in S}} \left( {I(x_{i} ;x_{s} ;C^{*} )} \right)} \right),$$

where, *I*(*x*_*i*_*;x*_*s*_;C^*^) denotes redundancy term. Shorting speaking and reader convenience, the complete steps of the proposed VMI is shown in Fig. 7.

**Figure 7:** Feature selection strategy form on VMI on electricity price.

## Modified honey bee mating optimization

In this section, the standard and developed model of the proposed algorithm is stated.

### Overview of standard HBMO

Here, HBMO was reviewed^84,85^,. The standard HBMO flowchart is shown in Fig. 8.

**Figure 8:** The standard HBMO algorithm, $d_{i}^{j} ,w_{i}^{j}$ and $b_{i}^{j}$ are *j*th gene of *i*th, worker and brood, respectively, *Sp*_*i*_ is *i*th individual in queen’s spermatheca, *β*_*HBMO*_ is generated in interval [0, 1], $\delta_{HBMO}$ is generated and $\varepsilon_{HBMO}$ is pre-defined.

### Proposed modified HBMO

Albeit the standard HBMO shown an effective performance, but its rapid converges to local optima is a drawback for exploration and exploitation. As shown for Fig. 8, coefficient *β*_*HBMO*_ was generated for interval [0, 1] which directly effects on global search and can’t guarantee its global solution.

However, in the modified HBMO, *β*_*HBMO*_ update equation is proposed by:

23 $$\beta_{i,j}^{t + 1} = \left\{ {\begin{array}{*{20}l} {\min \left( {1,\beta_{i,j}^{t} + (1 - \beta_{0} ) \times \exp \left( {\frac{{(d_{i,j}^{t + 1} - p_{i,j} )^{2} }}{{ - 2\sigma^{2} }}} \right) + \phi } \right),} \hfill & {{\text{if}}\{ \eta_{i} (t),\eta_{i} (t - 1)\} > 0} \hfill \\ {\max \left( {0.1,\beta_{i,j}^{t} - \beta_{0} \times \left( {1 - \exp \left( {\frac{{(d_{i,j}^{t + 1} - p_{i,j} )^{2} }}{{ - 2\sigma^{2} }}} \right)} \right) - \phi } \right),} \hfill & {{\text{if}}\{ \eta_{i} (t),\eta_{i} (t - 1)\} < 0} \hfill \\ {\beta_{i,j}^{t} ,} \hfill & {{\text{otherwise}}} \hfill \\ \end{array} } \right..$$

where $\beta_{i,j}^{t + 1}$ is a coefficient of the *j*th dimension of the *i*th drone or brood at iteration *t* + 1. $\beta_{0}$ is initial value for this coefficient, $\sigma$ refers to Gaussian kernel width, and it is calculated in each iteration to make better converge. $\phi$ is a small positive constant (0.001). $\eta_{i}$ dictates the *i*th drone to be succeed in the optimization process, which can be defined by:

24 $$\eta_{i} (t) = \left\{ {\begin{array}{*{20}c} 1 & {{\text{if fit(x}}_{i}^{t + 1} {\text{) < fit(p}}_{i} )} \\ { - 1} & {{\text{otherwise}}} \\ \end{array} } \right..$$

Moreover, employ chaotic operator in HBMO to enhance the local search. Chaotic sequences are simple and rapid to produce and memory, due to its features of unpredictability, non-periodic and ergodicity^102^. Therefore, we used the logistic equation as follows:

25 $$c_{k + 1}^{j} = \mu \times c_{k}^{j} + (1 - c_{k}^{j} ),\mu = 4,j = 1,2,...,N.$$

The $c_{k + 1}^{j}$ denotes *j*th chaos solution at iteration *k*.

## Proposed strategy of day-ahead electricity price forecasting

This section is organized as the following steps:

*Step 1* Set *A*_*i*_ as a threshold factor to make electricity price matrix for interval time *h* (*P*_*h*_) and training vector as follows:

26 $$I_{N} = \left[ {\begin{array}{*{20}c} {P_{h + 1} } & {P_{h + 2} } & {P_{h + 3} } & {\begin{array}{*{20}c} \cdots & {P_{{h + \upsilon_{i} }} } \\ \end{array} } \\ {P_{h + 2} } & {P_{h + 3} } & {P_{h + 4} } & {\begin{array}{*{20}c} \cdots & {P_{{h + 1 + \upsilon_{i} }} } \\ \end{array} } \\ {P_{h + 3} } & {P_{h + 4} } & {P_{h + 5} } & {\begin{array}{*{20}c} \cdots & {P_{{h + 2 + \upsilon_{i} }} } \\ \end{array} } \\ {\begin{array}{*{20}c} \vdots \\ {P_{{h + N - \upsilon_{i} }} } \\ \end{array} } & {\begin{array}{*{20}c} \vdots \\ {P_{{h + N - \upsilon_{i} + 1}} } \\ \end{array} } & {\begin{array}{*{20}c} \vdots \\ {P_{{h + N - \upsilon_{i} + 2}} } \\ \end{array} } & {\begin{array}{*{20}c} {\begin{array}{*{20}c} \ddots \\ \cdots \\ \end{array} } & {\begin{array}{*{20}c} \vdots \\ {P_{h + N} } \\ \end{array} } \\ \end{array} } \\ \end{array} } \right],T_{N} = \left[ \begin{gathered} P_{h + 1} \hfill \\ P_{h + 2} \hfill \\ P_{h + 3} \hfill \\ \vdots \hfill \\ P_{h + N} \hfill \\ \end{gathered} \right],$$

where subscript *N* denotes length of price history data. Thereafter, normalize *I*_*N*_ and *T*_*N*_ between 0 and 1.

*Step 2* To get all potential of proposed modified HBMO algorithm, the drone number, worker number, child number, queen’s spermatheca and maximum iteration are 50, 60, 30, 35 and 200, respectively. Note that these values obtained from solving different standard benchmarks and other papers which used HBMO.

*Step 3* Decompose electricity price signal in approximation (*A*_*i*_) and detail (*D*_*j*_) terms at level *i* and *j* by WPT tree, $W(p_{h} ;h = 1,...,T) = \{ a_{h} ,b_{h} ,c_{h} ,d_{h} ;h = 1,...,T\}$. To avoid the computational burden, the Shannon-Renyi entropy employed to select best branches.

*Step 4* As aforementioned illustration in step 3, considering detail and approximation into prediction framework with simultaneous form is a new contribution which rise the computational time. To make better way for learning part, VMI is applied for each candidate branches of WPT output. Resulting have best output vector {*x*_1_, *x*_2_,*…,* *x*_*n*_} to send for learning part.

*Step 5* The learning is main part of prediction. In other words, previous tools are tried to make a simple way for learning part based on valuable input data so as to decrease the forecasting error. However, if the learning part dose not be powerful to follow linear and nonlinear pattern, the WPT and VMI will not be useful lonely. The proposed LSSVM-SFK tries to make best performance in linear and nonlinear terms which shown in Fig. 9. The electricity price forecasts at day *D* needed to previous data to *D*-1. The electricity price at day *D* (24 h) are announced by Independent System Operator (ISO) for *D*-2.

**Figure 9:** Proposed time framework for price forecasting.

*Step 6* Calculate error-based objective function:

27 $$Obj = \frac{1}{N}\sum\limits_{i = 1}^{N} {\frac{{P_{i}^{f} - P_{i}^{a} }}{{P_{i}^{a} }}} ,$$

where, $P_{i}^{f}$ and $P_{i}^{a}$ denotes the forecast and actual price values, respectively.

*Step 7* Employ proposed modified HBMO algorithm to optimally set the LSSVM-SFK variables. In other words, proposed modified HBMO follows overall structure in Fig. 8 and objective function in Eq. (27) to decreases the prediction error. A typical close-loop flowchart is shown in Fig. 10.

**Figure 10:** A typical overview of relation between HBMO and learning method in order to decreases the prediction error.

*Step 8* Employ WPT to obtain price of day *D*, $W^{ - 1} (\{ a_{h}^{est} ,b_{h}^{est} ,c_{h}^{est} ,d_{h}^{est} ;h = T + 1,...,T + 24\} ) = P_{h}^{W,est}$, where superscript *est* denote estimated value in detail or approximation subseries.

*Step 9* Update HBMO coefficients and chaos population in order to discover the new possible solutions.

*Step 10* If the stop criterion is satisfy then print forecast result for day *D*, otherwise, go to step 2. The stop criteriosn in this study is number of iteration in HBMO algorithm.

## Results

Suggested model is evaluated on Spanish, New South Wales (NSW) (data is available at) and Hourly Ontario Energy Price (HOEP) (data is available at) as three well-known electricity markets^103–105^.

### Evaluating the forecasting error

This paper employs some error-based indices to make comparison with available methods. These indices are defined based on daily (*N* = 24 h) and weekly (*N* = 168 h) time periods. Shorting speaking, they can be formulated as follows:

Mean Absolute Percentage Error (MAPE):

28 $$MAPE_{day/week} = \frac{1}{N}\sum\limits_{i = 1}^{N} {\frac{{\left| {P_{i}^{f} - P_{i}^{a} } \right|}}{{P_{m} }}} ,$$

29 $$P_{m} = \frac{1}{N}\sum\limits_{i = 1}^{N} {P_{i}^{a} } .$$

Root Mean Square Error (FMSE):

30 $$RMSE_{day/week} = \sqrt {\frac{1}{N}\sum\limits_{i = 1}^{N} {\left( {P_{i}^{a} - P_{i}^{f} } \right)^{2} } } .$$

Median Error (MeE):

31 $$MeE_{day/week} = \frac{1}{N}\sum\limits_{i = 1}^{N} {\frac{{\left| {P_{i}^{a} - P_{i}^{f} } \right|}}{{\tilde{P}_{N} }}} ,$$

where $\tilde{P}_{N}$ is the median price for a specified period.

### Spanish electricity market

Since more of papers used this market to evaluate their forecasting algorithm, therefore, it will be reasonable to make a comprehensive compression with them in day-ahead electricity price forecasting. Firstly, input data are normalized between 0 and 1. It helps feature selection to make better decision in low space with least distance between valley and peak points in price signal. After it, the proposed WPT applied on input data to make corresponding sub-series, approximation and detail. The original Spanish electricity price is shown in top subplot of Fig. 11 and corresponding WT coefficients are shown in Fig. 11, also resulting of WPT is shown in Fig. 12. It is clear that WPT make better pattern compare to WT in noisy or residential term.

**Figure 11:** Appling of WT on Spanish electricity price with its coefficients and residential term.

**Figure 12:** Appling of WPT on Spanish electricity price with residential term, autocorrelation and FFT spectrum.

Then, the proposed VMI employed to chose best input data for minimum redundancy. In this regard, 49 days are selected as training data and one day considered as validated data, resulting have 50 days. To have comparison with other feature selection, resulting of Correlation Analysis (CA)^27^, MI^27^, GMI^35^ and proposed VMI are presented in Table 1.

**Table 1:** Selected features and proposed VMI methods for Spanish market.

Rank	CA^27^		MI^27^		GMI^35^		VMI	
	Selected feature	Value	Selected feature	Value	Selected feature	Value	Selected feature	Value
1	P_h-1_	0.92	P_h-168_	1.00	P_h-1_	0.91	P_h-24_	1.00
2	P_h-168_	0.85	P_h-1_	0.99	P_h-168_	0.91	P_h-48_	0.97
3	P_h-24_	0.83	P_h-336_	0.87	P_h-24_	0.88	P_h-1_	0.91
4	P_h-169_	0.79	P_h-672_	0.77	P_h-144_	0.86	P_h-72_	0.77
5	P_h-2_	0.79	P_h-167_	0.76	P_h-192_	0.86	P_h-23_	0.75
6	P_h-167_	0.79	P_h-337_	0.75	P_h-48_	0.86	P_h-25_	0.72
7	P_h-144_	0.78	P_h-169_	0.72	P_h-120_	0.85	P_h-96_	0.69
8	P_h-25_	0.78	P_h-504_	0.70	P_h-3_	0.85	P_h-47_	0.67
9	P_h-23_	0.77	P_h-673_	0.69	P_h-42_	0.84	P_h-49_	0.67
10	P_h-192_	0.77	P_h-144_	0.69	P_h-72_	0.84	P_h-120_	0.66
11	P_h-48_	0.76	P_h-24_	0.69	P_h-216_	0.84	P_h-192_	0.65
12	P_h-120_	0.75	P_h-312_	0.65	P_h-166_	0.84	P_h-144_	0.62
13	P_h-72_	0.73	P_h-216_	0.65	P_h-169_	0.84		
14	P_h-96_	0.73	P_h-192_	0.65	P_h-96_	0.84		
15	P_h-145_	0.73	P_h-335_	0.63				
16	P_h-193_	0.73	P_h-360_	0.61				
17	P_h-143_	0.72	P_h-288_	0.61				
18	P_h-191_	0.72	P_h-697_	0.61				
19	P_h-121_	0.71						
20	P_h-49_	0.71						
21	P_h-47_	0.71						
22	P_h-119_	0.69						
23	P_h-73_	0.69						
24	P_h-95_	0.69						
25	P_h-170_	0.68						
26	P_h-97_	0.67						
27	P_h-71_	0.67						

All results are normalized with respect to their minimum and maximum values and *P*_*h-T*_ shows selected price in hour *T*, columns 2, 4, 6 and 8 are selected features and columns 3, 5, 7 and 9 are their values, respectively.

As tabulated result in Table 1 and 1400 input data, filtering ratio for CA, MI, GMI and VMI are 51.85%, 77.78%, 100% and 116.16%, respectively. According to same input samples, it can be obvious that the VMI has better performance with higher filtering ratio. The numerical result based on MAPE index is reported in Table 2. This table consulates many methods to make a comprehensive comparison and to the reader convenience and avoid many number of references in this paper, all methods and their references can be found in Ref.^91^. Based on numerical results in Table 2, the numerical result are listed for 4 test weeks in year 2002^84^.

**Table 2:** MAPE of Spanish electricity market.

Method	Winter	Spring	Summer	Fall	Average
ARIMA, 2003^35^	6.32	6.36	13.39	13.78	9.96
Mixed-model, 2007^35^	6.15	4.46	14.90	11.68	9.30
NN, 2007^35^	5.23	5.36	11.40	13.65	8.91
Wavelet-ARIMA, 2005^35^	4.78	5.69	10.70	11.27	8.11
WNN, 2007^35^	5.15	4.34	10.89	11.83	8.05
FNN, 2006^35^	4.62	5.30	9.84	10.32	7.52
PSS, 2011^35^	5.98	4.51	9.11	10.07	7.42
HIS, 2009^35^	6.06	7.07	7.47	7.30	6.97
AWNN, 2008^35^	3.43	4.67	9.64	9.29	6.75
NNWT, 2010^35^	3.61	4.22	9.50	9.28	6.65
SRN, 2013^35^	4.11	4.37	9.09	8.66	6.56
RBFN, 2011^35^	4.27	4.58	6.76	7.35	5.74
CNEA, 2009^35^	4.88	4.65	5.79	5.96	5.32
CNN, 2009^35^	4.21	4.76	6.01	5.88	5.22
HNES, 2010^35^	4.28	4.39	6.53	5.37	5.14
MI + CNN, 2012^35^	4.51	4.28	6.47	5.27	5.13
WPA, 2011^35^	3.37	3.91	6.50	6.51	5.07
MI-MI + CNN, 2012^35^	4.29	4.20	6.31	5.01	4.95
WT-MI-SVM, 2014^35^	4.41	4.52	5.42	5.41	4.94
HEA, 2014^35^	3.04	3.33	5.38	4.97	4.18
WT-CLSSVM + EGARCH, 2013^35^	2.00	1.65	3.73	2.92	2.58
WT + ARIMA-CRACH, 2010^35^	0.63	0.65	1.19	2.18	1.16
WT + GMI + LSSVM-B + S-OLABC, 2016^35^	0.58	0.59	1.01	2.13	1.07
Proposed method	0.54	0.53	0.99	2.02	1.02

Furthermore to make comparison form on variance error, Table 3 listed variance for the forecasting errors for all methods. According to this index, result shows good performance. The forecasting algorithm has high accurate and robust in prediction than other methods in all seasons.

**Table 3:** Error variance of Spanish electricity market.

	Winter	Spring	Summer	Fall	Average
ARIMA, 2003	0.0034	0.0020	0.0158	0.0157	0.0092
NN, 2007	0.0017	0.0018	0.0109	0.0136	0.0070
Wavelet-ARIMA, 2005	0.0019	0.0025	0.0108	0.0103	0.0064
FNN, 2006	0.0018	0.0019	0.0092	0.0088	0.0054
AWNN, 2008	0.0012	0.0031	0.0074	0.0075	0.0048
NNWT, 2010	0.0009	0.0017	0.0074	0.0049	0.0037
HIS, 2009	0.0034	0.0049	0.0029	0.0031	0.0036
CNEA, 2009	0.0036	0.0027	0.0043	0.0039	0.0036
CNN, 2009	0.0014	0.0033	0.0045	0.0048	0.0035
RBFN, 2011	0.0015	0.0019	0.0047	0.0049	0.0033
WPA, 2011	0.0008	0.0013	0.0056	0.0033	0.0027
MI + CNN, 2012	0.0014	0.0014	0.0033	0.0022	0.0021
HNES, 2010	0.0013	0.0015	0.0033	0.0022	0.0021
MI-MI + CNN, 2012	0.0014	0.0014	0.0032	0.0023	0.0021
WT-MI-SVM, 2014	0.0017	0.0018	0.0087	0.0045	0.0041
HEA, 2014	0.0008	0.0011	0.0026	0.0014	0.0015
WT-CLSSVM + EGARCH, 2013	0.0002	0.0002	0.0012	0.0010	0.0007
WT-ARIMA + CRACH, 2010	0.0002	0.0002	0.0009	0.0008	0.0005
Proposed method	0.0001	0.0002	0.0006	0.0006	0.0003

Moreover, so as to a make graphical view for reader in day-ahead electricity price forecasting, Fig. 13 shows day-day and day-week electricity price forecasting based on the actual, forecast and forecast error signals.

**Figure 13:** Spring forecast (**A**) day, (**B**) week.

#### NSW electricity market

NSW was considered to day-ahead electricity price forecasting. Electricity market is more complicated than its predecessor, therefore, input data is given in year 2016. As mentioned in “Proposed Strategy of day-ahead electricity price forecasting” section, firstly all input data are normalized between 0 and 1, VMI is employed to get input. To make a comparison based on forecasting indices, three months are considered. The forecasting result via forecasting framework is compared to another models in Table 4. This comparison is based on feature selection, wavelet transform, learning algorithms and optimization algorithm. The forecasting framework is more powerful than other methods. Albeit, some obtained result from proposed forecasting framework and other methods are near but the proposed method is overlay better.

**Table 4:** MAPE for forecasting error of NSW.

Methods	April, 2016	July, 2016	October, 2016	January, 2017	Average
DWT + MI + SVM + HBMO	7.564	8.745	9.424	8.030	8.440
WPT + VMI + SVM + HBMO	5.093	6.948	8.093	6.780	6.728
DWT + MI + LSSVM + HBMO	4.536	4.771	7.094	5.764	5.541
WPT + VMI + LSSVM + HBMO	4.223	4.568	6.787	5.509	5.271
DWT + VMI + LSSVM-SFK + HBMO	4.995	5.092	6.216	5.348	5.412
WPT + VMI + LSSVM-SFK + HBMO	3.581	4.378	6.023	4.891	4.718
DWT + MI + SVM + Modified HBMO	5.837	6.983	8.342	7.093	7.063
WPT + VMI + SVM + Modified HBMO	4.825	5.719	7.389	6.012	5.986
DWT + MI + LSSVM + Modified HBMO	4.194	4.793	6.905	5.532	5.356
WPT + VMI + LSSVM + Modified HBMO	3.972	4.562	6.452	5.165	5.037
DWT + MI + LSSVM-SFK + Modified HBMO	3.562	4.247	6.021	4.783	4.653
WPT + VMI + LSSVM-SFK + Modified HBMO	3.421	4.093	5.783	4.621	4.479

For comparison and obtain view of day and week forecast accuracy, NSW data in year 2016 are presented in Fig. 14.

**Figure 14:** Data of NSW electricity market; (**A**) day, (**B**) week.

#### Hourly Ontario energy price (HOEP) electricity market

As the last case study to evaluate the proposed forecasting framework, the electricity market was choose. Electricity market clearing prices are planned every 5 min therefore it need more reliable forecast algorithm to efficiency capture the linear and nonlinear patterns. The effectiveness of the proposed forecasting framework is evaluated by Ontario’s electricity market over year 2016. The general simulation in this market procedure is similar to the both previous markets. For comparison, all proposed methods in Table 5 are selected and results were reported in Table 5.

**Table 5:** MAPE of forecasting error of electricity market.

Methods	April, 2016	July, 2016	October, 2016	January, 2017	Average
DWT + MI + SVM + HBMO	18.542	17.763	18.563	16.039	17.72
WPT + VMI + SVM + HBMO	16.262	16.095	17.534	15.832	16.43
DWT + MI + LSSVM + HBMO	16.093	15.734	17.221	15.009	16.01
WPT + VMI + LSSVM + HBMO	15.458	15.093	16.564	14.095	15.30
DWT + VMI + LSSVM-SFK + HBMO	15.054	14.635	16.032	13.655	14.84
WPT + VMI + LSSVM-SFK + HBMO	13.654	13.342	14.093	13.029	13.52
DWT + MI + SVM + Modified HBMO	13.452	13.027	13.985	12.675	13.28
WPT + VMI + SVM + Modified HBMO	13.102	12.894	13.673	12.043	12.92
DWT + MI + LSSVM + Modified HBMO	10.991	10.412	11.029	11.457	10.97
WPT + VMI + LSSVM + Modified HBMO	9.7864	8.5631	9.8753	10.652	9.71
DWT + MI + LSSVM-SFK + Modified HBMO	8.5643	7.0945	9.0921	8.6743	8.35
WPT + VMI + LSSVM-SFK + Modified HBMO	7.5362	6.0943	6.7384	5.9683	6.58

HOEP forecasts created in this paper has more accurate than other models and obtained error of the proposed above 22% is better than best of them, DWT + MI + LSSVM-SFK + Modified HBMO. DWT + MI + SVM + HBMO record worst data. For reader convince the electricity market data were presented in Fig. 15.

**Figure 15:** Electricity market data; (**A**) day, (**B**) week.

### Discussion on forecasting tools

In this section, the proposed algorithm is discussed and evaluated under various test functions, which are:

#### Modified HBMO converge

For comparison PSO, HBMO and suggested HBMO the Langermann's benchmark is examined^95^ and optimization problem is *x*_1_ and *x*_2_ and minima are obtained via:

32 $$\begin{gathered} f(x_{1} ,x_{2} ) = - \sum\limits_{i = 1}^{5} {\frac{{c_{i} \cos (\pi [(x_{1} - a_{i} )^{2} + (x_{2} - b_{i} )^{2} ])}}{{e^{{\frac{{(x_{1} - a_{i} )^{2} + (x_{2} - b_{i} )^{2} }}{\pi }}} }}} , \hfill \\ a = \left[ {\begin{array}{*{20}l} {\begin{array}{*{20}c} 3 & 5 & 2 & 1 \\ \end{array} } & 7 \\ \end{array} } \right]^{T} ,b = \left[ {\begin{array}{*{20}c} {\begin{array}{*{20}l} 5 & 2 & 1 & 4 \\ \end{array} } & 9 \\ \end{array} } \right]^{T} ,c = \left[ {\begin{array}{*{20}l} {\begin{array}{*{20}c} 1 & 2 & 5 & 2 \\ \end{array} } & 3 \\ \end{array} } \right]^{T} . \hfill \\ \end{gathered}$$

The data were reported in Table 6 and via applying improvement of HBMO, performance was increased.

**Table 6:** Convergence frequencies.

Method	Range of iteration					
	0–50	50–100	100–200	200–500	500–1000	> 1000
Modified HBMO	42	31	13	12	2	0
HBMO	24	18	30	18	8	2
PSO	4	14	26	33	12	11

In order to evaluate the performance of the proposed method in comparison with other methods, Table 7 shows the types of test functions and the results obtained are presented in Table 8. As shown in the results, the proposed method has performed better than other methods.

**Table 7:** The mathematical detailed of employed benchmark functions, *D* dimension, *[L,U]* lower and upper bands, *Fun* function name, *No* number, *Min* minimum value.

No	Fun	[L,U]	D	Formulation	Min
**Many local minima group**					
1	Ackley	[− 32, 32]	30	$f_{1} (x) = - 20\exp \left( { - 0.2\sqrt {\frac{1}{D}\sum\limits_{i = 1}^{D} {x_{i}^{2} } } } \right) - \exp \left( {\frac{1}{D}\sum\limits_{i = 1}^{D} {\cos (2\pi x_{i} )} } \right) + 20 + \exp (1)$	0
2	Bukin N. 6	$$\begin{gathered} x_{1} \in \left[ { - 15, - 5} \right] \hfill \\ x_{2} \in \left[ { - 3,3} \right] \hfill \\ \end{gathered}$$	2	$f_{2} (x) = 100\sqrt {\left| {x_{2} - 0.01x_{1}^{2} } \right|} + 0.01\left| {x_{1} + 10} \right|$	0
3	Cross-in-tray function	[− 10, 10]	2	$f_{3} (x) = - 0.0001\left( {\left| {\sin (x_{1} )\sin (x_{2} )\exp \left( {\left| {100 - \frac{{\sqrt {x_{1}^{2} + x_{2}^{2} } }}{\pi }} \right|} \right)} \right| + 1} \right)^{0.1}$	** − **2.06261
4	Drop-wave	[− 5.12, 5.12]	2	$f_{4} (x) = \frac{{1 + \cos \left( {12\sqrt {x_{1}^{2} + x_{2}^{2} } } \right)}}{{0.5\left( {x_{1}^{2} + x_{2}^{2} } \right) + 2}}$	− 1
5	Eggholder	[− 512, 512]	2	$f_{5} (x) = - (x_{2} + 47)\sin \left( {\sqrt {\left| {x_{2} + \frac{{x_{1} }}{2} + 47} \right|} } \right) - x_{1} \sin \left( {\sqrt {\left| {x_{1} - x_{2} - 47} \right|} } \right)$	− 959.6407

**Table 8:** Statistical results obtained different algorithms through 30 independent runs on mentioned benchmark functions, Best, Worst, Mean and STD denotes the best solution, the worst solution, the mean solution and the standard deviation, respectively.

No	Algorithms indices	GA	PSO	HBMO	GWO	Proposed
f_1_	Best	2.142E+00	7.053E−03	2.897E−03	1.065E-10	8.921E−012
	Worst	3.525E+00	1.279E−01	1.432E+00	4.873E−03	7.332E−010
	Mean	3.240E+00	9.858E−02	2.761E−02	7.565E−06	6.843E−011
	STD	3.058E−01	1.586E−02	1.076E−01	3.762E−02	7.154E−05
f_2_	Best	7.837E+01	5.381E+00	3.323E+00	2.546E−03	1.534E−05
	Worst	9.651E+02	9.043E+01	4.782E+00	4.726E−02	4.039E−05
	Mean	8.564E+01	7.542E+01	3.895E+00	1.657E−02	3.312E−05
	STD	1.243E+01	1.054E+01	2.746E+00	1.323E−01	5.625E−07
f_3_	Best	− 0.323E+00	− 0.645E+00	− 1.892E+00	− 1.997E+00	− 2.062E+00
	Worst	1.248E+00	1.121E+00	2.619E−01	− 1.143E+00	− 1.938E+00
	Mean	1.032E+00	0.342E+00	− 1.125E+00	− 1.657E+00	− 2.000E+00
	STD	8.637E+01	9.748E+00	3.524E−01	5.847E−02	3.827E−03
f_4_	Best	− 1.425E−01	− 4.837E−01	− 9.924E−01	− 1.000E+00	− 1.000E+00
	Worst	3.243E+00	− 1.093E−01	− 5.423E−01	− 7.837E−01	− 8.736E+00
	Mean	1.907E−01	− 1.623E−01	8.897E−01	− 8.879E−01	− 7.262E+00
	STD	1.783E+01	5.425E−01	1.029E−02	5.024E−03	1.323E−05
f_5_	Best	− 7.653E+02	− 9.321E+02	− 9.594E+02	− 9.596E+02	− 9.596E+02
	Worst	− 6.536E+02	− 9.025E+02	− 9.389E+02	− 9.563E+02	− 9.653E+02
	Mean	− 7.192E+02	− 9.294E+02	− 9.951E+02	− 9.578E+02	− 9.609E+02
	STD	3.201E+00	3.052E−01	1.443E−03	1.493E−04	3.32E−05

#### VMI analyze

In this section used Sonar data to evaluate the VMI performance comparing other well-known feature selection methods which this data can be found from Ref.. Table 9 denotes classifications rate via MLP to proposed via some models for data set^106^. It can be found from Table 6 that VMI outperformed all MIFS, MIFS-U and NMIFS^96^ for all number of candidate inputs. It can be concluded that VMI can consider both redundancy and relevancy. On the other hand, whole general information content is taken into account.

**Table 9:** Classifications for sonar data set.

No. inputs	NMIFS	mRMR	MIFS	MIFS-U	VMI
4	80.19	78.46	78.17	76.25	82.65
7	85.19	80.09	83.46	76.92	87.12
11	86.36	79.80	83.85	76.35	86.93
15	86.73	81.06	85.19	82.98	88.54

#### Effect of kernel fuzzy in learning

As last test system, Alpha and Delta data sets are selected which they are defined for the Large Scale Challenge. LSSVM-SFK and LSSVM series for 100,000 and 50,000 samples for training sets and Alpha and Delta are dense sets^107^. LSSVM-SFK need lower iterations than LSSVM to obtain same error in Fig. 16.

**Figure 16:** Test errors (in %), (**A**) number of epochs in LSSVM-SFK (Alpha data set), (**B**) training duration of LSSVM-SFK (Alpha data set), (**C**) number of epochs in LSSVM (Delta data set) and (**D**) training duration of LSSVM (Delta data set).

## Conclusions

To obtain high accuracy of electricity price forecasting, forecasting framework was suggested that was from WPT, VMI, and LSSVM-SFK by modified honey bee mating optimization (HBMO). The proposed framework is evaluated by Spanish data, NSW, and Ontario electricity markets. Superior of forecasting framework in electricity price is attributed to 3 parts. WPT is converted original price to subsets using high-pass and low-pass filters so as to obtain behaving signals. Next, VMI is calculated via historical price and low calculation CPU time. As final, modified HBMO method can tune appropriate control variables of the LSSVM-SFK model such as weight and bias, in which choosing unsuitable adjusting control variables leads to over- or under-fitting. The proposed day-ahead electricity price forecasting by hybrid framework is also compared to the available forecasting methods. The numerical result based on prediction error indices demonstrates that the proposed forecasting framework considerably improves the forecast accuracy in all electricity markets.
